# miR-135a-5p Suppresses TBK1 and Activates NRF2/TXNIP Antioxidant Pathway in LPS-Driven ALI in Mice

This article has been retracted.

**DOI:** 10.1155/2022/9088727

**Published:** 2022-07-20

**Authors:** Guotao Zou, Yiwen Zeng, Yingjuan Wang, Yong Luo

**Affiliations:** ^1^Department of Pediatrics, Yongchuan Hospital of Chongqing Medical University, 439 Xuanhua Road, Yongchuan District, Chongqing, China 402160; ^2^Department of Emergency, Yongchuan Hospital of Chongqing Medical University, 439 Xuanhua Road, Yongchuan District, Chongqing, China 402160

## Abstract

**Objective:**

Acute inflammation and oxidative stress are present in large numbers in patients with acute lung injury (ALI). This investigation probed miR-135a-5p/TBK1 axis within ALI together with its new therapeutic target.

**Methods:**

MLE-12 cultures were treated with lipopolysaccharide (LPS) and transfected with miR-135a-5p mimics or TBK1 vector. An ALI mouse model was also established. Analysis was done on the relationships between TBK1 and miR-135a-5p. Inflammatory components, SOD, MDA, and ROS content were all assessed.

**Results:**

Obvious inflammatory lesions were observed in lung tissues of ALI mice. Overexpression of miR-135a-5p or TBK1 knockdown remarkably decreased IL-1*β*, IL-6, and TNF-*α* serum concentrations and increased IL-10 level within lung tissues. Activated NRF2/TXNIP pathway and oxidative stress were additionally found within ALI murines, which were regulated by miR-315a-5p and TBK1. Further research revealed that miR-135a-5p negatively regulated TBK1 expression to mediate proinflammatory response and oxidative stress.

**Conclusion:**

miR-135a-5p targeted TBK1 to regulate inflammatory/oxidative stress responses in ALI. Such results might bring a new potential target for ALI treatment.

## 1. Introduction

Acute lung injury (ALI) is defined as a collection of acute hypoxemic respiratory failure accompanied with bilateral pulmonary infiltrations [1]. ALI can lead to a high morbidity up to 40% and has become a common and serious clinical syndrome in ICU department worldwide [2]. Despite recent advances in the treatment for ALI, the clinic outcomes and prognosis of ALI patients are rather poor [3]. Therefore, new treatments and novel therapeutic strategies for ALI are of great significance.

Acute lung injury (ALI) denotes a serious injury with an uncontrolled acute inflammatory response and activated oxidative stress, which ultimately leads to pulmonary endothelium and epithelial dysfunction [4]. The severity and development of the inflammatory response are thought to be related to the prognosis of ALI patients [5]. Meanwhile, a lot of data point to oxidative stress as a crucial factor in ALI development. Lipopolysaccharide- (LPS-) evoked ALI/ARDS model has been widely reported [6, 7]. A previous study revealed that Trillin attributed to the downregulation of MDA and inflammatory cytokines and the upregulation of CAT, SOD, GSH, and GSH-Px in ALI that were driven of LPS [8]. However, the underlying molecular mechanism for signaling pathways in inflammation and oxidative stress is still unclear.

Numerous studies have shown that microRNA (miR)-135a-5p is connected to autophagy and inflammatory response in a number of illnesses. According to a publication, miR-135a-5p overexpression or downregulation in atherosclerosis inhibits the ox-LDL-driven inflammatory response [9]. Another research indicated that miR-135a-5p inhibited oxidative stress/inflammatory response to restricted cerebral ischemia-reperfusion injury via regulating NR3C2 [10]. Similar result was also reported by Chen and Li in cerebral hypoxia/reoxygenation injury [11]. However, up to now, no studies focus parts played by miR-135a-5p within ALI.

miR-135a-5p's downstream target, TANK-binding kinase 1 (TBK1), plays a crucial part in numerous physiological pathways, including oxidative stress and inflammation [12]. According to a recent study, TBK1 is an endogenous inhibitor of RIPK1, and it also inhibits RIPK1-driven neuroinflammation and apoptosis during development and ageing [13]. However, in another study, Lin et al. revealed that overexpression of TBK1 activated NF-*κ*B activity, as well as MAPKs and Akt signaling pathway in osteoclast differentiation [14]. These studies indicate that TBK1 plays dual roles in inflammation of different diseases or bioprocesses. However, how TBK1 influences ALI is inadequately illustrated.

The following paragraphs describe how the paper is organised: Section 2 presents the research materials and methods. The experiments and findings are covered in Section 3. The discussion portion is included in Section 4. The research project is completed in Section 5.

### 1.1. Objective

In the current study, we wanted to investigate the molecular mechanisms underlying the miR-135a-5p/TBK1 axis inside ALI. Our results demonstrated that in LPS-driven mouse ALI, miR-135a-5p controlled inflammation and oxidative stress by targeting TBK1 and activating the NRF2/TXNIP antioxidant pathway. Such present research might be available novel research and therapeutic targets for ALI.

## 2. Methods

### 2.1. ALI Model Establishment and Animal Treatment

Forty-eight C57BL/6 (6-8 weeks with 18~20 g) male mice (Beijing Vital River Laboratory Animal Technology™ Co., Ltd.) were kept within standard cages with 50-70% of humidity at 24 ± 1°C. This study followed international guidelines for animal research projects and was accepted by the Animal Ethics Committee of YongChuan Hospital of ChongQing Medical University.

The establishment of ALI model was conducted as reported elsewhere [15]. In brief, mice were anesthetized with a 1 percent pentobarbital sodium, followed with a single intratracheal instillation dose of 0.05 mL *Escherichia coli* LPS (Sigma, Santa Clara, CA, USA) with dose of 5 mg/kg suspended in saline solution. The controls received the equal volume of saline solution.

For murine overexpression/inhibition of miR-135a-5p or TBK1, lentiviral plasmid-based miR-135a-5p mimic stable transfection was performed (Sigma-Aldrich, cat. no. MLMIR0048), as well as si-TBK1, pcDNA3.1-TBK1 (from GeneChem Corp., Shanghai, China, without sequence information), and corresponding NCs were injected into mice via tail vein (100 *μ*L, 2 × 10^7^ TU/mL). In all experiments, six animals were used in each group.

### 2.2. Hematoxylin and Eosin (HE) Staining

After the tests, the mice were slowly filled with an overdose of carbon dioxide gas before being put to death. The lung tissues were cut into three mm portions. After dehydrating the samples and fixing them in neutral formalin (10%), paraffin-embedded blocks were eventually produced. Briefly, the sections were immersed in xylene and alcohol, following with the staining with hematoxylin and eosin. Finally, histopathology observation was conducted using an optical microscope.

### 2.3. Cell Culture and Treatments

MLE-12 cells (ATCC) were grown within RPMI-1640 (Sigma-Aldrich) augmented using 10% FBS, 100 IU/mL penicillin and 100 *μ*g/mL streptomycin (Sigma-Aldrich™) within an incubator (37°C/5% CO_2_). For *in vitro* model, cultures were exposed to 10 *μ*g/mL LPS.

Regarding cell transfection, this was performed using miR-135a-5p mimics, pcDNA3.1-TBK1, or the counterpart NCs (5 nM) through Lipofectamine® 3000 (Invitrogen™, Waltham, MA, USA) within serum-free Opti-MEM® medium.

### 2.4. Western Blotting

This was performed in order to detect TBK1, Nrf2, and TXNIP. In brief, all proteomic content was collected from lung tissue/MLE-12 cultures and quantitated through the Pierce™ BCA Protein Assay Kit® (Thermo Scientific™). Subsequently, 20 *μ*g proteomic aliquots underwent SDS-PAGE and were transported onto PVDF which were consequently placed into incubation together with primary antibody (4°C overnight), and subsequent incubation with Goat Anti-Rabbit IgG H&L secondary antibody (ab96899, 1/1000) at 37°C for 45 min. Primary antibodies used were purchased from Abcam (USA): anti-TBK1 antibody (ab227182, 1/500), anti-Nrf2 antibody (ab92946, 1/1000), and anti-TXNIP antibody (ab188865, 1/1000). GAPDH served as internal/normalization control/reference.

### 2.5. Quantitative RT-PCR Analysis

miR-135a-5p/TBK1transcriptomic expression within tissue samples/MLE-12 cells was detected. First, total RNA was extracted from lung tissues and MLE-12 cells using the TRIzol® (Sigma-Aldrich™) method, and quantification was carried out with a NanoDrop spectrophotometer (ND-1000, ThermoFisher Scientific). Subsequently, the conversion from RNA into cDNA was performed through TransScript® one-step gDNA removal and cDNA Synthesis SuperMix kit (Applied Biosystems). For the detection of miRNA, a miRcute miRNA qPCR detection kit (SYBR Green) on a 7900 HT Sequence Detection System was conducted in PCR reactions. For the quantification of mRNA, SYBR GREEN Master Mix® (Thermo Fisher Scientific, Inc.™) over the ABI 7500® platform (Applied Biosystems) was performed. The primary primers were used in PCRs: TBK1 forward 5′-GGAGCCGTCCAATGCGTAT-3′, reverse 5′-GCCGTTCTCTCGGAGATGATTC-3′; miR-135a-5p forward 5′-AACCCTGCTCGCAGTATTTGAG-3′, reverse 5′-GCGGCAGTATGGCTTTTTATTCC-3′; U6 forward 5′-ACTCCTGCCACTAGAGCTTGT-3′, reverse 5′-CTCCGGGAACCAGCATTGTTA-3′; GAPDH forward 5′-AGGTCGGTGTGAACGGATTTG-3′, reverse 5′-GGGGTCGTTGATGGCAACA-3′. U6 and GAPDH served as the controls. mRNA expressions determined through 2^−ΔΔCt^ methodology.

### 2.6. Dual-Luciferase Reporter Assay

Prediction for bonding sequence across miR-135a-5p/TBK1 was conducted on using Starbase (http://starbase.sysu.edu.cn/) and TargetScan (http://www.targetscan.org); design of wild-type (WT) and mutant (MUT) fragments in TBK1 was performed accordingly. The WT and MUT of 3′-UTR of TBK1 sequences with/without the predicted binding responsive element for miR-135a-5p were amplified and subcloned to the p-MIR-report plasmid (Promega (Beijing) Biotech Co., Ltd. Beijing, China). Then, using Lipofectamine 3000, MLE-12 cells were cotransfected with miR-135a-5p vector (an inhibitor or mimic) and WT-TBK1 or MUT-TBK1 or NC vector (an inhibitor or mimic) (Invitrogen). MLE-12 cultures were extracted for detection using luciferase assay kits after two days of incubation (Promega™). Luciferase activities of cells was normalized using Renilla luciferase activities.

### 2.7. Enzyme-Linked Immunosorbent Assay (ELISA)

Serum levels for IL-6, IL-1*β*, TNF-*α*, and IL-10 were measured by ELISA assay. Blood samples of the mice were collected and detected using corresponding commercial ELISA kits: IL-1*β*Kit (#MBS175967), IL-6 Kit (#MBS2023471), IL-10 Kit (#MBS2021945), and TNF-*α* (#MBS175787, all from MyBioSource).

### 2.8. Measurement SOD, MDA, and ROS

Expression of SOD, ROS, and MDA in tissues and MLE-12 cells was detected using corresponding kits (Nanjing Jiancheng Bio-Technology™ Co., Ltd.) as instructed within manufacturer protocols.

### 2.9. Statistical Analysis

Continuous normally distributed datasets reflected mean ± SD. Comparative analyses across two groups performed through Student's *t*-test. Overall, *P* < 0.05 was deemed to confer statistical significance. SPSS 18.0® and GraphPad 6.0 were used for the analysis.

## 3. Result

In this section, we define the overexpressed miR-135a-5p or inhibited TBK1 attenuates inflammation-based responses within mice and LPS-driven ALI, overexpression of miR-135a-5p or inhibition of TBK1 activated NRF2/TXNIP antioxidant pathway and suppresses oxidative stress, and miR-135a-5p negatively regulates TBK1 expression in detail.

### 3.1. Overexpressed miR-135a-5p or Inhibited TBK1 Attenuates Inflammation-Based Responses within Mice and LPS-Driven ALI

This investigation initially probed miR-135a-5p/TBK1 role/s within LPS-driven ALI and inflammation-based responses within mice. Representative images of lung tissue in each group was shown in Figure 1(a). Obvious inflammation in LPS-driven lung specimens was observed, which was alleviated by miR-135a-5p mimics or si-TBK1. RT-qPCR/Western blotting analyses revealed an around 2-fold increase in miR-135a-5p expression following miR-135a-5p mimic transfection, with an approximately 2- to 3-fold decrease of TBK1 expression by si-TBK1 transfection in LPS-driven lung tissues; additionally, miR-135a-5p mimics suppressed TBK1 expression (Figure 1(b)). ELISA results revealed both miR-135a-5p mimics and si-TBK1 inhibited serum level for TNF-*α*, IL-1*β*, and IL-6 though elevated expression of IL-10 (Figure 1(c)). Such revelations indicated overexpression of miR-135a-5p or inhibition of TBK1 attenuated ALI and inflammation.

### 3.2. Overexpression of miR-135a-5p or Inhibition of TBK1 Activated NRF2/TXNIP Antioxidant Pathway and Suppresses Oxidative Stress

This investigation additionally probed regulating mechanistic/s for miR-135a-5p and TBK1 for NRF2/TXNIP signal pathway as well as oxidative stress. Protein expression of NRF2 and TXNIP was detected in each group. The findings showed that in the lung tissues of LPS-induced mice, TXNIP expression increased by about 3-fold whereas NRF2 expression decreased by around 4-fold. However, miR-135a-5p overexpression or inhibition of TBK1 increased NRF2 expression and decreased TXNIP expression (Figure 2(a)). We also noticed obvious elevation in MDA content and ROS generation and notable decline in SOD level in LPS-driven lung tissue. However, miR-135a-5p mimics or si-TBK1 remarkably inhibited the expression of MDA and ROS but enhanced SOD content (Figure 2(b)). These findings suggested overexpressed miR-135a-5p or inhibited TBK1 might activate NRF2/TXNIP antioxidant pathway and inhibit oxidative stress within LPS-driven ALI.

### 3.3. miR-135a-5p Mediates Inflammation and Oxidative Stress through Regulating TBK1 within Murine LPS-Driven ALI

Regulating mechanistic/s for miR-135a-5p within murine LPS-driven ALI inflammatory and oxidative stress responses were investigated. Dataset outcomes showed miR-135a-5p mimics aroused an approximately 3-fold reduction of TBK1, which was reversed by pcDNA3.1-TBK1 transfection in lung tissues (Figure 3(a)). Upregulated miR-135a-5p suppressed serum levels of proinflammatory factors but enhanced serum expression of anti-inflammatory interleukin, which was also rescued by upregulated pcDNA3.1-TBK1 (Figure 3(b)). Moreover, NRF2/TXNIP antioxidant pathway was activated by miR-135a-5p upregulation, reversing by overexpressed TBK1 (Figure 3(c)). Meanwhile, MDA content and ROS generation were inhibited, and the expression of SOD was enhanced by upregulated miR-135a-5p, rescued through overexpressed TBK1 in LPS-driven lung tissues (Figure 3(d)). The above results revealed miR-135a-5p-mediated inflammation and oxidative stress through regulating TBK1 in LPS-driven ALI in mice.

### 3.4. miR-135a-5p Negatively Regulates TBK1 Expression

In order to substantiate the regulation between TBK1/miR-135a-5p, MLE-12 mice cultures were used within this study. Firstly, the successful transfections of miR-135a-5p vector (inhibitor/mimics) were proven in MLE-12 cells (Figure 4(a)). Based on bioinformatics analysis, bonding location for miR-135a-5p/TBK1 was forecasted (Figure 4(b)). A dual-luciferase reporter test revealed that miR-135a-5p overexpression lowered the fluorescence intensity of TBK1-WT by a factor of 1.5 whereas miR-135a-5p knockdown increased it by about 3-fold. No obvious effects by miR-135a-5p upon TBK1-MUT were observed (Figure 4(c)). RT-qPCR analysis suggested negatively regulating miR-135a-5p influence upon TBK1, further verified in Western blotting analysis (Figures 4(d) and 4(e)). The result confirmed miR-135a-5p bound to TBK1 with negative regulation for TBK1 expression.

### 3.5. miR-135a-5p Mediates Inflammation and Oxidative Stress through Regulating TBK1 within LPS-Driven MLE-12 Cultures

Finally, molecular control by miR-135a-5p/TBK1 upon oxidative stress and inflammation-based responses within LPS-driven MLE-12 cultures was investigated. pcDNA3.1-TBK1 increased TBK1 expression by 4 times within MLE-12 cultures (Figure 5(a)). miR-135a-5p mimics suppressed TBK1 expression, which was rescued by cotransfection of pcDNA3.1-TBK1. Besides, overexpressed miR-135a-5p downregulated TNF-*α*, IL-6, and IL-1*β* and enhanced IL-10. Meanwhile, overexpressed TBK1 reversed the regulation of miR-135a-5p on inflammatory response (Figure 5(b)). It was also revealed that NRF2/TXNIP pathway was triggered by overexpressed miR-135a-5p, but was rescued by upregulated TBK1 (Figure 5(c)). Overexpression of miR-135a-5p decreased MDA and ROS expression while increasing SOD levels. Overexpression of TBK1 reversed this effect. The results supported miR-135a-5p-mediated oxidative stress and inflammatory responses through regulating TBK1 within LPS-driven MLE-12 cells.

## 4. Discussion

ALI brings huge burden to the critically ill patients with high mortality and morbidity [16]. As we know, inflammation and oxidative stress have pivotal parts within ALI pathogenesis/development [17, 18]; nevertheless, the underlying mechanism remains uncertain. This *in vitro and in vivo* study investigated the regulating miR-135a-5p influence over LPS-driven ALI. Such findings demonstrate that miR-135a-5p mediates oxidative stress and inflammation through regulating TBK1 in LPS-driven ALI.

miR-135a-5p exhibits anti-inflammatory influence across multiple diseases. As reported, suppressing miR-135a-5p attenuated neuropathic pain by the inhibition of autophagy and inflammatory response in CCI rat model [19]. In addition, miR-135a-5p showed an inhibitory effect on the activation of NLRP3 inflammasome, causing a suppression for neuronal autophagy and ischemic brain injury. Overexpression of miR-135a-5p increased cell proliferation but restrained cell apoptosis and the protein expressions associated with autophagy in neuronal cells [20]. Another study also found the suppression of miR-135a-5p/CXCL12/JAK-STAT signaling axis restrained inflammatory response and cell apoptosis in myocardial infarction, thereby alleviating myocardial injury [21]. However, no research illustrated the regulating parts played by miR-135a-5p within ALI. This study confirmed miR-135a-5p downregulation within ALI and that overexpressed miR-135a-5p could attenuate acute lung injury, inflammatory response as well as oxidative stress. Besides, miR-135a-5p mediated inflammation and oxidative stress through regulating TBK1 in lung injury.

TBK1 was reported to play anti-inflammatory roles in several studies. A recent research indicated TBK1 attenuated inflammation by phosphorylating and inducing the degradation of the IKK kinase NIK and negatively regulated NF-*κ*B expression through AMPK pathway in controlling metabolism [22]. However, more studies suggested TBK1 might activate inflammatory pathways during inflammation. Ahmad et al. demonstrated that TBK1 and IKKe were involved in the activation of IFN-inducing IFN-regulatory factor (IRF) transcription factors [23]. These inconsistent results indicated TBK1 might play a dual role in inflammatory response in different diseases. TBK1 is also found to be involved in affecting oxidative stress. Huh et al. reported TBK1 loss inhibited fasting-driven fatty acid oxidation in the liver [24]. Another study also revealed the inhibition of TBK1 alleviated lung injury, attenuated oxidative damage, and decreased expression of inflammatory factors in both mice and RAW264.7 mouse macrophages [25]. Nevertheless, the effect of TBK1 in acute lung injury has not been revealed in previous researches. This study illustrated that TBK1 inhibition not only suppressed inflammation and oxidative stress but also activated NRF2/TXNIP antioxidant pathway in lung injury.

## 5. Conclusion

In summary, our research revealed that overexpressed miR-135a-5p or inhibited TBK1 attenuated acute lung injury and inflammation, as well as activated NRF2/TXNIP antioxidant pathway and suppressed oxidative stress. Furthermore, we showed for the first time that miR-135a-5p reduced oxidative stress and inflammation by targeting TBK1 in MLE-12 cells. The findings could lead to the development of new treatment targets for acute lung injury in clinical settings.

## Figures and Tables

**Figure 1:** Overexpressed miR-135a-5p or inhibited TBK1 attenuates LPS-driven ALI and inflammatory response in mice. (a) Representative histopathological examination of mouse lung tissues by HE staining in LPS-driven group, LPS-driven group transfected with miR-135a-5p mimics, LPS-driven group transfected with si-TBK1, and corresponding NCs and the healthy controls. Scale bars: 25 *μ*m, magnified 400x, *n* = 6 for each group. (b) Expression of miR-135a-5p by qRT-PCR. (c) mRNA of TBK1 was determined through RT-qPCR, and TBK1 proteomic content was evaluated using Western blotting. (d) IL-1*β*, IL-6, TNF-*α*, and IL-10 levels were determined through ELISA kits. *P* values were assessed through Student's *t* test.

**Figure 2:** Overexpressed miR-135a-5p or inhibited TBK1 activated NRF2/TXNIP antioxidant pathway and suppresses oxidative stress. (a) NRF2/TXNIP proteomic levels were analyzed through western blotting. (b) MDA, ROS, and SOD of LPS-driven lung tissues were analyzed using ELISA kits. *P* values were assessed through Student's *t* test.

**Figure 3:** miR-135a-5p mediates inflammation and oxidative stress through regulating TBK1 in LPS-driven murine ALI. (a) mRNAs for miR-135a-5p and TBK1 were determined through RT-qPCR, and protein level for TBK1 was evaluated using Western blotting in lung tissues in LPS-driven group, LPS-driven group transfected with miR-135a-5p mimics, LPS-driven group transfected with miR-135a-5p mimics and pcDNA3.1-TBK1, and the corresponding NC controls. (b) Levels of IL-1*β*, IL-6, TNF-*α*, and IL-10 were determined using ELISA kits. (c) Protein levels of NRF2 and TXNIP were detected using Western blotting. (d) MDA, ROS, and SOD of LPS-driven lung tissues were analyzed using ELISA kits. *P* values were assessed through Student's *t* test.

**Figure 4:** miR-135a-5p negatively regulates TBK1 expression. (a) miR-135a-5p transfected efficiency was analyzed using qRT-PCR. (b) Biding site between miR-135a-5p and TBK1 was predicted by Starbase (http://starbase.sysu.edu.cn/) and TargetScan (http://www.Targetscan.org/). (c) Targeting relationship between miR-135a-5p and TBK1 was analyzed by dual-luciferase reporter assay. (d, e) mRNA and protein levels of TBK1 were detected using qRT-PCR and Western blotting. *P* values were assessed through Student's *t* test.

**Figure 5:** miR-135a-5p mediates inflammation and oxidative stress through regulating TBK1 in LPS-driven MLE-12 cells. (a) Transfection efficiency of TBK1 was confirmed using qRT-PCR. (b) Expression of miR-135a-5p by qRT-PCR. (c) mRNA and protein levels of TBK1 were detected using qRT-PCR or Western blotting in LPS-driven MLE-12 cells, LPS-driven MLE-12 cells transfected with miR-135a-5p mimics, LPS-driven MLE-12 cells transfected with miR-135a-5p mimics and pcDNA3.1-TBK1, and the corresponding NC controls. (d) Serums IL-1*β*, IL-6, TNF-*α*, and IL-10 were determined using ELISA kits. (e) Supernatant protein levels of NRF2 and TXNIP were detected using Western blotting. (f) Supernatant contents of MDA, ROS, and SOD were determined using ELISA kits. *P* values were assessed through Student's *t* test.

## Data Availability

All data can be obtained from the manuscript or from request to the author.
